The article "Neuropathological and neuroprotective features of vitamin B12 on the dorsal spinal ganglion of rats after the experimental crush of sciatic nerve: an experimental study" was retracted in 2016. Reasons: misconduct by an author; plagiarized text; compromised peer review; false authorship.

# Neuropathological and neuroprotective features of vitamin B_12_ on the dorsal spinal ganglion of rats after the experimental crush of sciatic nerve: an experimental study

**DOI:** 10.1186/1746-1596-8-123

**Published:** 2013-07-31

**Authors:** Rahim Hobbenaghi, Javad Javanbakht, Ehan Hosseini, Shahin Mohammadi, Mojtaba Rajabian, Pedram Moayeri, Mehdi Aghamohammad hassan

**Affiliations:** 1 Department of Pathology, Faculty of Veterinary Medicine, University of Urmia, Urmia, Iran; 2 Department of Pathology, Faculty of Veterinary Medicine, University of Tehran, Tehran, Iran; 3 Faculty of Para Veterinary Medicine, Ilam University, Ilam, Iran; 4 Graduate Faculty of Veterinary Medicine, University of Urmia, Urmia, Iran; 5 Food Hygiene Department, University of Shahekord, Shahekord, Iran; 6 Resident of Large Animal Internal Medicine Department, University of Shahekord, Shahekord, Iran; 7 Department of Clinical Science, Faculty of Veterinary Medicine, University of Tehran, Tehran, Iran

**Keywords:** Dorsal root ganglion, Rat, Surgery, Sciatic nerve, Vitamin B_12_

## Abstract

**Background:**

Spinal motoneuron neuroprotection by vitaminB12 was previously reported; the present study was carried out to evaluate neuroprotectivity in the dorsal root ganglion sensory neuron.

**Methods:**

In present study thirty-six Wister-Albino rats (aged 8–9 weeks and weighing 200–250 g) were tested. The animals were randomly divided into 6 groups which every group contained 6 rats. Group A: received normal saline (for 42 days); Group B: vitamin B12 was administered (0.5 mg/kg/day for 21 days); Group C: received vitamin B12 (1 mg/kg/day for 21days); Group D: received vitamin B12 (0.5 mg/kg/day for 42 days); Group E; received vitamin B12 (1 mg/kg/day for 42 days); Group F; received no treatment. The L5 Dorsal Root Ganglion (DRG) neurons count compared to the number of left and right neurons .Furthermore, DRG sensory neurons for regeneration were evaluated 21 or 42 days after injury (each group was analyzed by One-Way ANOVA test).

**Results:**

(1): The comparison of left crushed neurons (LCN) number with right non-crushed neurons in all experimental groups (B, C, D and C), indicating a significant decline in their neurons enumeration (*p*<0/05). (2): The comparison of test group’s LCN with the control group’s LCN revealed a significant rise in the number of experimental group neurons (*p*<0/05). (3): Moreover, comparing the number of right neurons in experimental groups with the number of neurons in crushed neurons indicated that the average number of right neurons showed a significant increase in experimental groups (*p*<0/05).

**Conclusion:**

Consequently, the probability of nerve regeneration will be increased by the increment of the administered drug dosage and duration. On the other hand, the regeneration and healing in Dorsal Spinal Ganglion will be improved by increase of administration time and vitamin B12 dose, indicating that such vitamin was able to progress recovery process of peripheral nerves damage in experimental rats. Finally, our results have important implications for elucidating the mechanisms of nerve regeneration. Moreover, the results showed that vitaminB12 had a proliferative effect on the dorsal root ganglion sensory neuron.

The article "Neuropathological and neuroprotective features of vitamin B12 on the dorsal spinal ganglion of rats after the experimental crush of sciatic nerve: an experimental study" was retracted in 2016. Reasons: misconduct by an author; plagiarized text; compromised peer review; false authorship.

**Virtual slides:**

The virtual slide(s) for this article can be found here: http://www.diagnosticpathology.diagnomx.eu/vs/7395141841009256

## Background

Unlike the central nervous system (CNS), neurons the peripheral nervous system (PNS) can regenerate by its own after physical injury because of activation of the intrinsic growth capacity of neurons [1].

The sciatic nerve, innervating the hind paw of the rat, is frequently used to study peripheral nerve regeneration. After crush injury, the fibers distal to the lesion undergo Wallerian degeneration: the axon and myelin degenerate and are ingested by Schwann cells and invading macrophages. Schwann cells surrounding the distal fibers proliferate so that the endoneurial tubes surrounding the original nerve fibers remain intact, providing the environment through which the regenerating axons can grow [2,3].

Peripheral nerve injury results in a loss of sensory and motor function and nerve repair often results in poor functional recovery. This is, in part, due to dorsal root ganglion (DRG) cell death, regeneration errors or failure to regenerate [4-6].

The sciatic nerve, comprising a mixed population of motor and sensory axons, is a commonly used model for studying nerve regeneration and it regeneration is accompanied by a variety of changes in the DRG neurons cell bodies and regeneration is associated with the expression of new genes and proteins [2,7].

The DRG consists of heterogeneous population of neurons. During development neurons must receive appropriate neurotrophic support to survive which is achieved by establishing appropriate peripheral target connections via their neuritis [8].

Injury to DRG neuron cellular body or central axon results in somatosensory defects that do not recover spontaneously. Lost DRG neurons are not replaced. Central axon response to injury is weak [9-11], leading to slow axonal regrowth [12], Moreover, the proximal and distal axonal processes of sensory neurons exhibit different regeneration rates: Dorsal root axons regenerate at a lower rate as compared to distal axon regrowth into the lesioned spinal or sciatic nerve [12-15]. The reasons for this discrepancy are not clear. The sensory neurons extending into the sciatic nerve are located in the L4–L6 dorsal root ganglion (DRGs). After sciatic nerve injury (SNI), the damaged neurons suffer important changes to switch the neuro-transmitter state to a pro-regenerative state [16].

The article "Neuropathological and neuroprotective features of vitamin B12 on the dorsal spinal ganglion of rats after the experimental crush of sciatic nerve: an experimental study" was retracted in 2016. Reasons: misconduct by an author; plagiarized text; compromised peer review; false authorship.

B-vitamins were reported to attenuate degenerating processes in the nervous system and therefore have been clinically administered in a combination of B_1_ (thiamine), B_6_ (pyridoxine), and B_12_ (cobalamine;Cbl)[17]. Ganglion count in rat after SNI Vitamin B12(vit B_12_) is a micronutrient that plays significant roles in numerous biological processes. It acts as a coenzyme, which is required for metabolism of folate and biosynthesis of nucleotide [18]. It helps maintaining normal functions of the brain. vit B_12_deficient neuropathy is well established in humans, and has also been described in animal models [19]. The CNS and especially the spinal cord are severely damaged by vit B_12_deficiency [20].

Vit B_12_ is transported in the blood bound to transcobalamin (TC) and internalized into cells by its receptor, (TC-R, also named CD320). In the cells, vit B_12_ is transferred to the cytoplasm by the lysosomal membrane vit B_12_ transporter (LMBRD1) and serves as cofactor for methyl malonylCoA mutase (Mut) and methionine synthase (MS) [21]. Futhermore, vit B_12_ deficiency leads to methionine deficiency, which is required for the synthesis of both phospholipids and myelin. In addition, vitamin B12 has been shown to exert antioxidant properties [22], which result from direct and indirect effects [23].

In parallel of this research several studies regarding vit B_12_ effects on nerves healing have been conducted. Yagihashi et al. (1982) suggested that continuous treatment with CH3-B12 had an ameliorative effect on the peripheral nerve lesions in experimental diabetic neuropathy [24]. In addition, Okada et al. (2010) showed that vit B_12_may provide a basis for more beneficial treatments of nervous disorders through effective systemic or local delivery of high doses of methylcobalamin to target organs [25]. Watanabe in 1994 tested a high dosage of vit B_12_ (500 mg/kg) on repairing the damaged nerves of rats, somehow the potential return of muscles action was significantly faster than that recorded in control group, which treated with high dose of vitamin B12, rats [26]. Swett et al. have studied on neurons dorsal root ganglion count in rat after SNI [27].

In the present study, we investigated the neuroprotective effects of vit B_12_on dorsal spinal ganglion of rats after the experimental sciatic nerve crush.

The article "Neuropathological and neuroprotective features of vitamin B12 on the dorsal spinal ganglion of rats after the experimental crush of sciatic nerve: an experimental study" was retracted in 2016. Reasons: misconduct by an author; plagiarized text; compromised peer review; false authorship.

## Methods

### Animals

All experimental protocols were approved by the local animal care committee in accordance with Faculty of Urmia Veterinary Medicine office regulations. In current study, 36 Wister-albino rats of both sexes, weighing 200–250 g, with averagely 6 weeks old were selected. The animals were kept two by two in individual propylene cages under standard laboratory conditions by the dimensions of 30×50×25 cm^3^. Rats were maintained on a 12 hour light/dark cycle at 22±1°C and 50±10% humidity. The animals were kept in standard room conditions and fed with standard rat diet and water ad libitum.

### Experimental protocol

The rats were divided into six groups and randomly allotted into one of six experimental groups each group contained six animals. Control animals in group A received normal saline (for 42 days) (n=6), and test animals in group B received vit B_12_following surgery (0.5 mg/kg/day for 21 days) (n=6); however, test animals of group C received vit B_12_following surgery (1 mg/kg/day for 21 days) (n=6). Test animals in group D received vit B_12_following surgery (0.5 mg/kg/day for 42 days) (n=6), whereas test animals in group E received vit B_12_following surgery (1 mg/kg/day for 42 days) (n=6), and in F: Sham group had no surgery and vit B_12_injection, and were euthanized after 42 days (n=6) in order to necropsy examination. In addition, the vit B_12_in experimental group was injected intraperitoneally.

### Surgical technique

DRG of the spinal cord segment L5 which mainly sciatic nerve is originated from is located in L1 vertebral column of the rat. Therefore, to remove it, according to the method of the mentioned article, spinal segment, dorsal root and related ganglion were removed from L1 of the vertebral column [28]. All of the operations were performed under microscope by same surgeon. The left lateral thigh was operated after shaving and preparing the skin with 10% povidone iodine. The sciatic nerve was exposed by opening the fascial plane between the gluteal and femoral musculature via a longitudinal incision (2–3 cm). All surgical procedures were carried out under ketamine hydrochloride (75 mg /kg) and Xylazine hydrochloride (5 mg/kg) anesthetic solutions, the sciatic nerve of such 30 rats was exposed at mid-thigh level and either crushed for 5 minutes with a pair of hemostatic forceps (9–10 mm size). Subsequently, the muscles and skin were separately sutured by 4/0 catgut thread and allowed to breathe room air. The surgery was followed by the animals’ special care until recovery.

### Sample collection and microscopic examination

In both group animals (the control and experimental), the left sciatic nerve had been crushed before the treatment was started and then sutured. The animals were anaesthetized with IP injection of sodium thiopenthal after 21 and 42 days. The left and right dorsal root ganglia-L5 and sections from distal parts of the right (non-operated) and left (operated) sciatic nerves were collected, fixed, and prepared for light microscopic examination. A 10 mm-long sample of the right sciatic nerve segment was removed without any injury, fixed, and prepared for histopathological examination. Tissue fragments were fixed in 10% neutral buffered formalin solution (for 72 hours), upon stability embedded in paraffin, sectioned at 5 μm thickness and stained with hematoxylin and eosin (H&E).

The article "Neuropathological and neuroprotective features of vitamin B12 on the dorsal spinal ganglion of rats after the experimental crush of sciatic nerve: an experimental study" was retracted in 2016. Reasons: misconduct by an author; plagiarized text; compromised peer review; false authorship.

### Method of calculating the number of neurons

To determine the total number of neurons in the spinal dorsal root node, the researchers used series of cross-sectional counting method. In this method, through examination of each neuronal population the sensory neurons, one of every 5 or 10 sections, were counted and the total cells were multiplied by 5 or 10, respectively to give an estimate of total cell numbers and neurons, containing clear nuclear or nucleus were counted. Finally, the total number of neurons in the dorsal root node was compared to that of different groups. The neuronal counting method was explained by Clarke [29]. Briefly, the left and right L5 DRG were removed and post-fixed in 4% paraformaldehyde then 30% sucrose, both at 4°C for 24 h. the ganglia were blocked in tissue freezing medium and stored at −80°C. Each entire ganglion was cut into serial 15-μm cryosections and 1 from 4 sections mounted onto gelatin-coated glass slides and dried overnight. Neuron counts were performed using light microscopy. By a camera (DP11 camera) mounted on top of the microscope, images from the sections were prepared at magnifications of ×100, ×400, and ×1000, normal and clear neuronal nuclei or nucleus were counted. Neuron loss was calculated by subtracting the number of neurons in ipsilateral ganglion from that in their contralateral controls. Loss was then expressed as a percentage of the neuron count in the control ganglia.

### Statistical analysis

The data were expressed as mean ± standard deviation (SD), and analyzed by repeated measures of variance. In order to comparing number of counted neurons between different groups a one-way ANOVA test and to evaluate time interventions and drug dosage, Duncan test were used. Experimental results were considered to be significantly different from control values with p-value set at.05 (SPSS).

## Results

The procedures for reconstructing the regenerated DRG neuron populations were identical to those used in an earlier study, describing the normal sciatic DRG neuron populations in the rat [30].

The article "Neuropathological and neuroprotective features of vitamin B12 on the dorsal spinal ganglion of rats after the experimental crush of sciatic nerve: an experimental study" was retracted in 2016. Reasons: misconduct by an author; plagiarized text; compromised peer review; false authorship.

The results of the present study indicated that there was a significant decrease in the number of DRG neurons in all groups with SNI compared to early stages of injury of the sham and control groups.

Furthermore, the results of this study demonstrated that compared to the number of neurons in left ganglions of crushing sciatic nerve (LGCSN) with neurons in right ganglions of non-crushing sciatic nerve (RGNCSN) in all experimental groups (EGs) (0/5 and 1 mg/kg, 21 and 42 days) a significant decrease in the number of EGs neurons was recorded (*p*<0/05). This decrease was 7015± 132 to 6336± 142 respectively (*p*<0/05) (Table 1).

**Table 1:** Indicates of the average number of neurons of left crushing sciatic nerve of all groups (A) compared to the right non-crushing sciatic nerve of the same groups (B)

**Groups**	**Mean ±SD A decrease in the number of neurons of A group in relation to B and their comparison with sham group**
21-day (0.5 mg/kg)	7015± 132
21-day (1 mg/kg)	7002± 109
42-day (0.5 mg/kg)	6749± 124
42-day (1 mg/kg)	6336± 142
Sham	8815± 114

Values are means ± SD (n=5). p<0.05 comparison to sham group.

Moreover, comparison the number of neurons in LGCSN (of each EG) with neurons in same side of the control group (CG) (*p*<0/05) revealed a significant increase in the frequency of EG neurons (*p*<0/05). The increase was 7079± 102 to7779± 123 respectively (*p*<0/05) (Table 2).

**Table 2:** Indicates of the average increase in the number of neurons of left crushing sciatic nerve of experimental group (A) compared to the right non-crushing sciatic nerve of the control group (B)

**Groups**	**Mean ±SD An increase in the number of neurons of A group in relation to B and their comparison with control group**
21-day (0.5 mg/kg)	7079± 102
21-day (1 mg/kg)	7069± 117
42-day (0.5 mg/kg)	7435± 200
42-day (1 mg/kg)	7779± 123
Control	7025± 173

Values are means ± SD (n=5). p=<0.05 comparison to the right non-crushing sciatic nerve of the control group.

On the other hand, comparison the number of right neurons in EGs with the number of neurons in CG indicated a significant increase in the average number of right EGs neurons (*p*<0/05). This increase was 7023± 164 to 7095± 171 respectively (*p*<0/05) (Table 3).

**Table 3:** Indicates of the average increase in the number of neurons of right non-crushing sciatic nerve of the experimental group (A) compared to the non-crushing sciatic nerve of the control group (B)

**Groups**	**Mean ±SD An increase in the number of neurons of A group in relation to B**
21-day (0.5 mg/kg)	7023± 164
21-day (1 mg/kg)	7028± 163
42-day (0.5 mg/kg)	7447± 119
42-day (1 mg/kg)	7095± 171

Values are means ± SD (n=4). p<0.05 comparison to the non-crushing sciatic nerve of the control group.

The article "Neuropathological and neuroprotective features of vitamin B12 on the dorsal spinal ganglion of rats after the experimental crush of sciatic nerve: an experimental study" was retracted in 2016. Reasons: misconduct by an author; plagiarized text; compromised peer review; false authorship.

In the treatment groups (0.5 mg/kg, 21 days) the number of DRG neurons after SNI revealed a significant rise in the number of neurons compared to that of the CG (*p*<0.05). Also the same significant difference was available in the number of neurons in other treatment groups (1 mg/kg, 21 days) (*p*<0.05). The comparison between two experimental 21-day groups of 0.5 mg/kg and 1 mg/kg showed no significant difference.

Additionally, in the treatment group (1 mg/kg, 42 days), the numbers of neurons solely demonstrated significant rise in comparison with CG (*p*<0.05). The number of neurons between 42-day group (0.5 mg/kg) and CG did not show remarkable increase. In addition, there was not any significant difference in 0.5 and 1 mg/kg 42-day groups (Figure 1).

**Figure 1:** **Histopathological evaluation of dorsal Root Ganglion neurons in the treatment and control groups. A**: Death of dorsal Root Ganglion (DRG) neurons in the control group that treated with normal saline, there were not nucleolus and nuclei (arrow), (H&G, x400). **B**: Note that of dorsal Root Ganglion (DRG) neurons in the experimental groups that treated vitamins B12, there were nucleolus and nuclei (arrow), (H&Gx400).

In order to investigate whether the neuroprotective effect of vit B_12_ is dose-dependent, we administered one higher dose of the vitamin (i.e., 1 mg/kg vit B_12_) 42 d after SNI surgery. As shown in Figure 2B, higher doses of the vitamin alleviated the neuroprotective behavior more effectively than lower doses (compare to Figure 2A), and stronger effects were again observed after the second drug injection which was given 24 h after the first injection. Thus, SNI-induced neuroprotective behavior was dose-dependently inhibited by systemic administration of vitamins B_12_.

**Figure 2:** Investigation neuron increase and decrease percentage in experiment groups compared to the right ganglions of non-crushing sciatic nerve and control group.

In order to examining the impact and simultaneous interaction of both factors (time and treatment dosage) in the number of neurons, a two-way ANOVA and Duncan test were used. The comparison between the control groups at 21 days after surgery represented a significant difference with treatment groups both in 21 and 42 days treatment groups. On the other hand, the number of neurons in control groups at 42 days after surgery was similar the number of neurons at 21-day groups for both dosages. The results indicated that neuron injury begins to repair 42 days after surgery while vit B_12_ accelerated such process conspicuously.

The article "Neuropathological and neuroprotective features of vitamin B12 on the dorsal spinal ganglion of rats after the experimental crush of sciatic nerve: an experimental study" was retracted in 2016. Reasons: misconduct by an author; plagiarized text; compromised peer review; false authorship.

## Discussion

Peripheral nerve regeneration is a complex biological process involving interactions among multiple cells, neurotrophic factors and extracellular matrice proteins [31]. This report led us to believe that a systemic examination of DRG neuron responses to vit B_12_ is advantageous to better understand the role of vitamin B12 in peripheral nerve regeneration.

The present study evaluated the protective effects of vit B_12_on the number of DRG cells recovery after inducing SNI in the rats.

In a serious trauma like SNI, a short period of localized ischemia is followed by evident increase in the pressure of endoneural fluid and defect of the normal capillary blood flow in the endoneurium [32]. Subsequently, Wallerian degeneration may arise distal to the lesion [14,17]. It has been shown that sciatic nerve crush leads to histological changes in the DRG cells number [33]. Loss of the neurons occurs and the nerve cells become less after peripheral nerve injury in the DRG [15,18]. This finding is in accordance with our results in which we showed the number of the cells were decreased.

Histological changes, such as decrease in the number of DRG cells after SNI, have been reported by other researchers [34-36]. Our results are in accordance with these findings, in which we demonstrated that the total number of L5-DRG cells after SNI were decreased.

Vit B_12_is also a good scavenger of the reactive oxygen species and is suggested to be a good neuroprotectant. It can pass through the blood brain barrier, which is an evidence of amplification of its neuroprotectant potential in neurodegenerative disorders such as Parkinson's and Alzheimer's diseases [37]. In addition, it has been reported that vit B_12_ has protective effects after spinal cord injuries. The previous studies have stressed the anti-apoptotic and anti*-*necrotic effects of the vit B_12_ on the neurons [38]. These reports may explain the beneficial effects of vit B_12_ in the present study after SNI. These properties including anti-inflammatory, antioxidant, anti-apoptotic and anti*-*necrotic might be effective in the present study.

In previous reports on the effects of vit B_12_ on neurons *in vivo*, high levels of vit B_12_ improved nerve conduction and regeneration in streptozotocin-diabetic rats [17], and experimental acrylamide neuropathy [26]. We used a rat SNI model in the present study to evaluate the effects of vit B_12_*in vivo*. However, we used continuous administration of doses of vit B_12_ (0.5 and 1 mg/kg/day) higher than that used in previous reports (500 μg/kg/day). Our morphological and histological evaluation offers a possible explanation of this phenomenon. Vit B_12_increased the regeneration of axons.

The article "Neuropathological and neuroprotective features of vitamin B12 on the dorsal spinal ganglion of rats after the experimental crush of sciatic nerve: an experimental study" was retracted in 2016. Reasons: misconduct by an author; plagiarized text; compromised peer review; false authorship.

We consider that repair discrepancy is due to the differences in the doses of vit B_12_and time of administration. In our study, vit B_12_had not remarkable affect on neurons at low*-*dose concentrations, especially with low-dose administration or short time, because the concentration of vit B_12_declines immediately [39] and the absorption of vit B_12_from the ileum and entire intestine is regulated by limitation of binding to gastric intrinsic factor and passive diffusion [40,41]. From the results of our study, we consider that it is necessary to devise new clinical methods, such as high-dose systemic or long time, to deliver high doses of vit B_12_ to target organs to treat nervous disorders more effectively. Thus, the high-dose vit B_12_ treatment together with long time might have the potential to treat not only peripheral nerve injury but also central nervous injury.

The results of our study indicated that the experimental groups, under treatment with vit B_12_, were prevented from reducing the number of neurons in DRG (Table. 2). Moreover, the DRG neurons decrease of left side of the operated experimental group compared to non-operated right side of the same group was slightly, especially it reached to the lowest degree (6336± 142) in 1mg/kg dosage in 42-day, and the result was significant compared to the other groups (p<0/05). On the other hand, the left neurons of 0/5mg/kg group in 21-day shows an increase of 7779± 123 compared to the same ganglion of the control group.

Also, according to Table 3, the neuronal mean increase shows a significant rise in association with the increase of vit B_12_ dosage and time that such variation in 0/5 and1 mg/kg group reached to 7023± 164 to 7095± 171respectively (Table 3). In addition, the decrease in the neurons death percentage of the right side of the non-crushing sciatic nerves compared to the same side of the control group was 20/32, 20/27, 20/05 and 19/51 percent (Table 3 and Figure 1 ).

On the other hand, the regeneration and healing in Dorsal Spinal Ganglion will be improved by increase of administration time and vit B_12_ dose, indicating that such vitamin was able to progress recovery process of peripheral nerves damage in experimental rats.

In parallel with our research several studies have been conducted. Yamatsu evaluated the effect of vitaminB12 on the nerve repair after a crush injury. Vit B_12_ demonstrated significant increase in the regeneration and improvement on SNI tests suggesting an inhibitory effect on the nerve degeneration and facilitating the regeneration after an injury [42]. Okada et al. evaluated the effectiveness of vit B_12_ on nerve regeneration and found that it demonstrated the greatest improvement on nerve regeneration [25]. Yamazaki also demonstrated that vit B_12_ improves the neuromuscular junction by decreasing nerve degeneration and improving nerve regeneration in the motor nerve terminals in a gracile axonal dystrophy mice model [43].

The article "Neuropathological and neuroprotective features of vitamin B12 on the dorsal spinal ganglion of rats after the experimental crush of sciatic nerve: an experimental study" was retracted in 2016. Reasons: misconduct by an author; plagiarized text; compromised peer review; false authorship.

In addition to, the results of this study confirm the results of one-way ANOVA and represent that the neurons construction and repairing started by time passage. Because the average number of neurons in under-prescription groups by vit B_12_ in 0.5mg/Kg and 1mg/Kg doses increased in 42-day experimental groups from 7435± 200 to7779± 123, and this difference was obvious and significant between the control group and 42-day experimental group in 1mg/kg dosage (p<0/05). In agreement with our study, Yagihushi et al., 1976 suggested that a constant 16-week cures by vit B_12_ (500 microgram/kg) had a completely repairing effect on the injured peripheral nerves in experimental diabetic neuropathy of rats. In another study, Taniguchi et al., 1987 indicated that vit B_12_ cured neuropathy in uromicina patients. They advised that vitamin B12 could be used as a cure in such forms of neuropathy [44]. In addition, another study by, Hasegawa et al. (1978) studies showed that the vitamin B complex facilitated functional recovery from nerve injury faster than its components, and showed that B1 and B12 had significant facilitating effects on the functional recovery as well [45].

In this study, we showed that the vitamin B12 was the most effective in promoting neuronal survival in DRG neurons. These results suggest that the metabolic pathway of vit B_12_, is associated with neuronal survival, but further understanding of this role and development of an effective delivery system for vitamin B12 may enable us to treat several nervous disorders and to obtain new insights into nerve regeneration.

## Conclusion

Our study suggests that vitamin B12 has neuroprotective and restorative effects on secondary pathochemical events after sciatic nerve injury in rats. These restorative effects have been mainly observed on neuronal numbers. We believe that further preclinical research into the utility of Cbl may indicate its usefulness as a potential treatment on neurodegeneration after trauma in rats but more and detailed experimental studies are needed to determine the effects of Cbl on the detrimental results of secondary sciatic nerve injury in human and animal. Furthermore, this study revealed that the regeneration and healing in Dorsal Spinal Ganglion will be improved by increase of administration time and vitamin B12 dose, indicating that such vitamin was able to progress recovery process of peripheral nerves damage in experimental rats.

The article "Neuropathological and neuroprotective features of vitamin B12 on the dorsal spinal ganglion of rats after the experimental crush of sciatic nerve: an experimental study" was retracted in 2016. Reasons: misconduct by an author; plagiarized text; compromised peer review; false authorship.

## Competing interests

The authors declare that they have no conflict of interest.

## Authors’ contributions

RH and SHM participated in the neurohistopathological evaluation, performed the literature review, acquired photomicrographs and drafted the manuscript and gave the final histopathological diagnosis. JJ performed sequencing alignment and manuscript writing .EH, MR,PM and MAMH edited the manuscript and made required changes. All authors have read and approved the final manuscript.
